The article "Efficacy of Glucocorticoid plus Intravenous Immunoglobulin in Children with Immunoglobulin-Insensitive Kawasaki Disease" was retracted in 2023. Reasons: signs of a paper mill; suspected computer-generated content; unreliable results or conclusions; concerns about the data.

# Efficacy of Glucocorticoid plus Intravenous Immunoglobulin in Children with Immunoglobulin-Insensitive Kawasaki Disease

**DOI:** 10.1155/2022/9011259

**Published:** 2022-04-13

**Authors:** Yongmei Ma, Jingjing Zhang, Rong Fan

**Affiliations:** ^1^Department of Child Immunology and Endocrinology, Baoji Maternal and Child Health Hospital, Baoji 721000, Shaanxi, China; ^2^Department of Pediatrics, Xijing Hospital, The First Affiliated Hospital of Air Force Military Medical University, Xi'an 710032, Shaanxi, China

## Abstract

This study mainly analyzes the clinical effect of glucocorticoid (GC) plus intravenous immunoglobulin (IVIG) in treating children with immunoglobulin (Ig)-insensitive Kawasaki disease (KD). From September 2013 to November 2021, 86 Ig-insensitive KD children were selected, including 46 children (observation group, Obs) treated with GC plus IVIG, and 40 children (control group, Con) treated with IVIG. The symptom (fever and fever) resolution time, inflammatory factors (C-reactive protein, CRP; procalcitonin, PCT; interleukin-6, IL-6), immune indicators (CD3^+^, CD4^+^, CD8^+^ T lymphocytes CD3^+^, CD4^+^, and CD4^+^/CD8^+^), and incidence of adverse reactions were compared between the groups. The results identified shorter fever and rash resolution time in Obs compared with Con. The posttreatment CRP, PCT, IL-6, and CD8^+^ and the incidence of adverse events reduced notably in Obs and were lower than Con, while CD3^+^, CD4^+^, and CD4^+^/CD8^+^ elevated statistically and were higher than that of Con. Our results indicate that GC plus IVIG can significantly promote symptom resolution, alleviate inflammatory response, and improve immune function in children with Ig-insensitivity KD, with favorable safety and clinical promotion value.

## 1. Introduction

Kawasaki disease (KD), a mucocutaneous lymph node syndrome named after its discoverer (Kawasaki), is an acute febrile inflammatory disease that tends to occur among infants and children [1, 2]. KD is the most common cause of acquired heart disease in children in developed countries and even leads to coronary artery aneurysms (CAA), elevating the risk of coronary artery thrombosis in the later stage [3]. In addition, the main clinical presentations of KD include persistent fever, pleural rash, conjunctival congestion, oral mucosal lesions, swollen neck lymph nodes, and severe hand swelling, which seriously threaten children's physical and mental health [4]. Although the diagnosis and treatment strategies of KD are constantly optimized, the clinical effects still leave much to be desired [5]. At present, the etiology and pathogenesis of the disease have yet to be clarified. Some studies have confirmed that it is related to the body's inflammatory microenvironment and immune dysfunction, which is mainly manifested as host immune dysregulation under inflammatory stimulation, and even activation of a series of immune-related cell groups including T lymphocyte groups in the acute phase of the disease [6]. Interestingly, in this regard, various intelligent diagnostic systems for improved heart disease diagnosis were also developed as it is most common in KD patients, which can facilitate the researchers towards KD treatment [7, 8]. It would be great if we could start from the pathogenesis of KD to find a more ideal and reliable treatment method, which will help improve the efficacy of KD children, reduce the risk of adverse events, and ease the public health burden related to KD.

The article "Efficacy of Glucocorticoid plus Intravenous Immunoglobulin in Children with Immunoglobulin-Insensitive Kawasaki Disease" was retracted in 2023. Reasons: signs of a paper mill; suspected computer-generated content; unreliable results or conclusions; concerns about the data.

Immunoglobulin (Ig), a regulator of the inflammatory process and immune response, is also vital in the effective connection between adaptability and the innate immune system [9]. Intravenous immunoglobulin (IVIG) has also been proved to be one of the standard treatments for KD, which can not only suppress inflammatory reactions through various regulatory mechanisms but also prevent the activation of innate immune cells [10]. However, some children with KD did not respond to IVIG treatment, which brings great challenges to disease treatment [11]. Glucocorticoid (GC) is a final product activated by the hypothalamus-pituitary-adrenal axis used to treat inflammation and autoimmune diseases and can regulate the cardiovascular tone, immune system, metabolism, and other physiological functions [12]. Besides, it can be used as a combination therapy with IVIG for myasthenia gravis in children with proven efficacy [13]. Previous studies have shown that GC plus IVIG is also applicable to treat acute KD, significantly shortening the fever time of children and inhibiting cytokines such as interleukin (IL)-2, IL-6, and IL-8 [14].

Given the current lack of research on the combined use of GC and IVIG in children with Ig-insensitive KD, we conduct related research to provide new clues for the treatment of this type of patient population.

## 2. Data and Methods

### 2.1. Baseline Data

From September 2013 to November 2021, 86 children with Ig-insensitivity KD were selected and assigned to an observation group (Obs; *n* = 46) and the control group (Con; *n* = 40) based on different therapies (GC plus IVIG and IVIG alone, respectively). The male-to-female and the mean age in Obs were 32 : 14 and (6.18 ± 1.12) years, respectively, while the data in Con were 28 : 12 and (5.85 ± 1.03) years. The two cohorts of patients exhibited no evident difference in baseline data like gender and age (*p* > 0.05; Table 1). This study is a retrospective study approved by the Ethics Committee of the Baoji Maternal and Child Health Hospital. The informed consent was signed by the patient's parent or guardian.

The article "Efficacy of Glucocorticoid plus Intravenous Immunoglobulin in Children with Immunoglobulin-Insensitive Kawasaki Disease" was retracted in 2023. Reasons: signs of a paper mill; suspected computer-generated content; unreliable results or conclusions; concerns about the data.

### 2.2. Eligibility Criteria

Inclusion criteria: meeting the diagnostic criteria for Ig-insensitive KD [15], ≤10 years old, normal cognitive and communication skills, no history of drug allergy, and no medication that may affect the results of this study within the past six months.

Exclusion criteria: presence of IVIG or GC contraindications, hematological system disorders or congenital diseases, organ dysfunction such as cardiac and hepatorenal dysfunction, and malignant tumors or infectious diseases.

### 2.3. Drug Treatments

Both groups were given oral aspirin (10–15 mg/kg, 3 times/day), and the dose was reduced to 3–5 mg/kg per day when fever subsided. On this basis, Con was given IVIG therapy, 1 g/kg per day for 15 days. Obs was additionally treated with GC based on the control group. Methylprednisolone sodium succinate (3–5 mg/kg/d) was injected intravenously for 30 min each time, once a day. After three consecutive days of treatment, it was changed to oral administration. The course of treatment was 15 days.

### 2.4. Measurement Indicators

Symptom resolution time: we mainly recorded the fever and rash resolution time of the two groups of children.

Inflammatory factors: we collected 5 mL of fasting cubital venous blood from both groups the next morning before and after treatment. After serum separation, enzyme-linked immunosorbent assay (ELISA) [16] was used to measure C-reactive protein (CRP), procalcitonin (PCT), and IL-6 in children following the operation steps of ELISA kits.

Immune indices: T lymphocytes (CD3^+^, CD4^+^, CD8^+^, and CD4^+^/CD8^+^) of children were detected by flow cytometry, and the experimental operation strictly followed the instrument instructions.

Incidence of adverse reactions (ARs): we mainly observed, recorded, and statistically analyzed the number of cases of adverse events such as nausea and vomiting, diarrhea, rash, dizziness and headache, renal function injury, and thromboembolic diseases in the two groups.

### 2.5. Statistical Processing

We used SPSS software (IBM Inc., version 17.0) for statistical analysis and exported the images through the GraphPad Prism software (version 6.0). The chi-square test (*χ*^2^) was utilized for comparisons of categorical data expressed as several cases/percentages (*n*/%) in the two groups. The intergroup and intragroup (before and after treatment) comparisons of continuous data represented by mean ± SEM were made using the independent samples *t*-test and paired *t*-test, respectively. *P* values less than 0.05 were considered statistically significant.

The article "Efficacy of Glucocorticoid plus Intravenous Immunoglobulin in Children with Immunoglobulin-Insensitive Kawasaki Disease" was retracted in 2023. Reasons: signs of a paper mill; suspected computer-generated content; unreliable results or conclusions; concerns about the data.

## 3. Results

### 3.1. Baseline Information

We analyzed children's general data and determined that the two arms were comparable (*p* > 0.05). The results were as follows: significant differences were absent between the groups in terms of sex, average age, time from disease onset to hospital admission, duration of fever, coronary artery disease, acute fever, rash, mucosal congestion, cardiovascular system damage, and family history (*p* > 0.05), as given in Table 1.

### 3.2. Impact of GC plus IVIG on Symptom Resolution Time

Fever and rash resolution time in Obs was observed as (1.22 ± 0.19) d and (2.53 ± 0.51) d, respectively. While, the data in Con was found to be (5.42 ± 1.24) d and (6.93 ± 1.51) d. Fever and rash resolution time was shorter in Obs than that of Con (Figure 1).

### 3.3. Impact of GC plus IVIG on Inflammatory Factors in Children

We detected and compared inflammatory factors CRP, PCT, and IL-6 between groups to evaluate the influence of the two treatments on children's inflammatory responses. The data showed no significant difference in inflammatory indexes between groups before treatment (*p* > 0.05). While, the posttreatment levels of the above inflammatory factors decreased in both groups (*p* < 0.05), with notably lower parameters in Obs (*p* < 0.05) (Figure 2).

### 3.4. Impacts of GC plus IVIG on Immune Function of Children

We compared the effects of the two treatment methods on children's immune function by detecting T lymphocytes before and after treatment. The data revealed no evident difference in T lymphocytes between the groups before treatment (*p* > 0.05). After treatment, CD3^+^, CD4^+^, and CD4^+^/CD8^+^ increased (*p* < 0.05), while CD8^+^ decreased (*p* < 0.05), with significant differences in T lymphocytes between the groups (*p* < 0.05) (Figure 3).

### 3.5. Impacts of GC plus IVIG on ARs in Children

In Obs, nausea, vomiting, rash, dizziness, and headache mainly occurred in 1 case each, and the incidence of ARs was 6.51%. In Con, there were 3 cases of dizziness and headache, followed by nausea, vomiting, diarrhea, and rash with 2 cases each, with an incidence of ARs of 22.50%. The incidence of ARs was lower in Obs than in Con (*p* < 0.05) (Table 2).

## 4. Discussion

KD is a self-limiting systemic vasculitis that can cause multiorgan arteritis, resulting in impaired multiple organ function [17]. Its incidence rate is still increasing, especially among men and children of Asian races [18]. This study mainly discusses the clinical effects of GC and IVIG in Ig-insensitive KD, aiming at contributing to the treatment of the disease.

The article "Efficacy of Glucocorticoid plus Intravenous Immunoglobulin in Children with Immunoglobulin-Insensitive Kawasaki Disease" was retracted in 2023. Reasons: signs of a paper mill; suspected computer-generated content; unreliable results or conclusions; concerns about the data.

In this study, we included 86 Ig-insensitive KD children and intervened with either the combination therapy of GC and IVIG (Obs) or IVIG monotherapy (Con). Our research results showed that the combined treatment had a remarkable effect on resolving the symptoms of fever and rash in children, suggesting that the combined intervention is more conducive to the clinical symptoms of children. IVIG preparations are composed of polyclonal plasma-derived IgG from thousands of donors, which secrete a large number of antibodies that are specific and conducive to play an anti-inflammatory role [19–21]. In KD, IVIG can reverse the abnormally delayed apoptosis of circulating neutrophils via lowering the blood neutrophil count [22]. At present, IVIG has been widely used in childhood diseases such as Guillain–Barre syndrome, Henoch–Schönlein purpura, and multiple-system inflammatory syndrome, exerting positive effects on relieving inflammation and clinical symptoms to varying degrees [23–25]. The antifever effect of GC has also been confirmed in infantile influenza, which can alleviate fever symptoms by inhibiting the secretion of proinflammatory cytokines [26]. It is known that in the acute stage of KD, the immune system will be activated, and excessive secretion of proinflammatory cytokines in circulation will be induced, leading to local and systemic injuries [27]. In the evaluation of inflammation, our data showed that the combination therapy significantly inhibited inflammatory indexes such as CRP, PCT, and IL-6, with more obvious inhibition than the monotherapy. This shows that the combined action of GC and IVIG is more effective in alleviating the inflammatory reaction of children. In terms of immune function, a more obvious improvement of T lymphocytes was observed in Obs, suggesting that the combined treatment can validly improve the immune function of children. Finally, we evaluated the safety of the two treatments and determined a higher safety profile in children treated with GC plus IVIG, which was manifested in a lower incidence of adverse events.

This study has confirmed the efficacy and safety of GC plus IVIG in treating children with Ig-insensitive KD, which can significantly resolve clinical symptoms, alleviate inflammation, and improve the immune function of children. However, this research still has potential limitations, which need to be gradually addressed in future research. First of all, the sample size of the study is small, and increasing the sample size will be more beneficial for the accuracy of the results. Second, if follow-up can be supplemented for prognostic analysis, the impact of the combined treatment on the prognosis of children with Ig-insensitive KD can be further evaluated. Finally, the underlying mechanism of their therapeutic effect can be further elucidated if the relevant basic research of combination therapy can be supplemented and their therapeutic mechanism in Ig-insensitive KD can be explored.

The article "Efficacy of Glucocorticoid plus Intravenous Immunoglobulin in Children with Immunoglobulin-Insensitive Kawasaki Disease" was retracted in 2023. Reasons: signs of a paper mill; suspected computer-generated content; unreliable results or conclusions; concerns about the data.

## 5. Conclusion

Here, we demonstrated the effect of the combined therapy of GC and IVIG in children with Ig-insensitive KD, and the results revealed that the combined therapy of GC and IVIG exhibited a remarkable effect for resolving the clinical symptoms of fever and rash in children. Additionally, in terms of inflammation, combination therapy significantly inhibited inflammatory indexes such as CRP, PCT, and IL-6, with more obvious inhibition than monotherapy. The combined treatment of GC and IVIG validly improve the immune function of children by causing significant improvement in T lymphocytes. Hence, this study suggests that GC plus IVIG has satisfactory clinical effects in treating children with Ig-insensitive KD, which can resolve the clinical symptoms, inflammatory reaction, and immune function of children to varying degrees, with certain safety, providing a new understanding for the treatment of such children.

## Figures and Tables

**Figure 1:** Effect of glucocorticoid combined with IVIG on symptom resolution time in children. (a) Comparison of fever resolution time between two groups. (b) Comparison of rash resolution time between two groups. ^*∗∗*^*P* < 0.01.

**Figure 2:** Effect of glucocorticoid combined with IVIG on inflammatory factors in children. (a) Comparison of CRP between two groups of children. (b) Comparison of PCT between two groups of children. (c) Comparison of IL-6 between two groups of children. ^*∗∗*^*P* < 0.01.

**Figure 3:** Effect of glucocorticoid combined with IVIG on immune function of children. (a) Comparison of CD3^+^ between two groups of children. (b) Comparison of CD4^+^ between two groups of children. (c) Comparison of CD8^+^ between two groups of children. (d) Comparison of CD4^+^/CD8^+^ between two groups of children. ^*∗∗*^*P* < 0.01.

**Table 1:** General information of children in the two groups (*n* (%), mean ± SD).

Variables	*n*	Control group (*n* = 40)	Observation group (*n* = 46)	Statistics (*χ*^2^ or *t*)	*P*
Gender				0.002	0.965
Male	60	28 (70.00)	32 (69.57)		
Female	26	12 (30.00)	14 (30.43)		
Average age (years)	86	5.85 ± 1.03	6.18 ± 1.12	1.414	0.161
Time from disease onset to hospital admission (d)	86	6.68 ± 1.49	6.54 ± 1.14	0.493	0.624
Duration of fever (d)	86	3.66 ± 0.71	3.74 ± 0.77	0.498	0.620
Coronary artery disease				0.089	0.765
No	61	29 (72.50)	32 (69.57)		
Yes	25	11 (27.50)	14 (30.43)		
Acute fever				0.024	0.877
No	33	15 (37.50)	18 (39.13)		
Yes	53	25 (62.50)	28 (60.87)		
Rash				0.040	0.841
No	42	20 (50.00)	22 (47.83)		
Yes	44	20 (50.00)	24 (52.17)		
Mucosal hyperemia				0.013	0.911
No	50	23 (57.50)	27 (58.70)		
Yes	36	17 (42.50)	19 (41.30)		
Cardiovascular system damage				0.055	0.815
No	57	26 (65.00)	31 (67.39)		
Yes	29	14 (35.00)	15 (32.61)		
Family medical history				0.050	0.823
No	57	27 (67.50)	30 (65.22)		
Yes	29	13 (32.50)	16 (34.78)		

The article "Efficacy of Glucocorticoid plus Intravenous Immunoglobulin in Children with Immunoglobulin-Insensitive Kawasaki Disease" was retracted in 2023. Reasons: signs of a paper mill; suspected computer-generated content; unreliable results or conclusions; concerns about the data.

**Table 2:** Effect of glucocorticoid combined with IVIG on adverse events in children (*n* (%)).

Categories	Control group (*n* = 40)	Observation group (*n* = 46)	*χ* ^2^ value	*P* value
Nausea and vomiting	2 (5.00)	1 (2.17)	—	—
Diarrhea	2 (5.00)	0 (0.00)	—	—
Rash	2 (5.00)	1 (2.17)	—	-
Dizziness and headache	3 (7.50)	1 (2.17)	—	-
Renal function injury	0 (0.00)	0 (0.00)	—	—
Thrombosis disease	0 (0.00)	0 (0.00)	—	—
Total	9 (22.50)	3 (6.51)	4.549	0.033

## Data Availability

The data used to support the findings of this study are available from the corresponding author upon request.
